# Berberine Suppresses Stemness and Tumorigenicity of Colorectal Cancer Stem-Like Cells by Inhibiting m^6^A Methylation

**DOI:** 10.3389/fonc.2021.775418

**Published:** 2021-11-15

**Authors:** Ziyi Zhao, Jinhao Zeng, Qiang Guo, Kunming Pu, Yi Yang, Nianzhi Chen, Gang Zhang, Maoyuan Zhao, Qiao Zheng, Jianyuan Tang, Qiongying Hu

**Affiliations:** ^1^ Traditional Chinese Medicine (TCM) Regulating Metabolic Diseases Key Laboratory of Sichuan Province, Chengdu, China; ^2^ Hospital of Chengdu University of Traditional Chinese Medicine, Chengdu, China; ^3^ Geriatric Department, Traditional Chinese Medicine (TCM) Regulating Metabolic Diseases Key Laboratory of Sichuan Province, Chengdu, China; ^4^ Department of Geriatrics, Chengdu First People’s Hospital, Chengdu, China; ^5^ Department of Ultrasound, the Second People’s Hospital of Chengdu, Chengdu, China; ^6^ Chengdu Women’s and Children’s Central Hospital, School of Medicine, University of Electronic Science and Technology of China, Chengdu, China; ^7^ Department of Laboratory Medicine, Hospital of Chengdu University of Traditional Chinese Medicine, Chengdu, China

**Keywords:** cancer stem-like cells (CSCs), Berberine, m6A methylation, β-catenin, FTO

## Abstract

**Background:**

Cancer stem cells (CSCs) are able to survive after cancer therapies, resulting in tumor progression and recurrence, as is seen in colorectal cancer. Therapies targeting CSCs are regarded as novel and promising strategies for efficiently eradicating tumors. Berberine, an isoquinoline alkaloid extracted from the Chinese herbal medicine Coptis chinensis, was found to have antitumor activities against colorectal cancer, without knowing whether it exerts inhibitory effects on colorectal CSCs and the potential mechanisms.

**Methods:**

In this study, we examined the inhibitory roles of Berberine on CSCs derived from HCT116 and HT29 by culturing in serum-free medium. We also examined the effects of Berberine on m^6^A methylation *via* regulating fat mass and obesity-associated protein (FTO), by downregulating β-catenin.

**Results:**

We examined the effects of Berberine on the tumorigenicity, growth, and stemness of colorectal cancer stem-like cells. The regulatory effect of Berberine on N6-methyladenosine (m^6^A), an abundant mRNA modification, was also examined. Berberine treatment decreased cell proliferation by decreasing cyclin D1 and increasing p27 and p21 and subsequently induced cell cycle arrest at the G_1_/G_0_ phase. Berberine treatment also decreased colony formation and induced apoptosis. Berberine treatment transcriptionally increased FTO and thus decreased m^6^A methylation, which was reversed by both FTO knockdown and the addition of the FTO inhibitor FB23-2. Berberine induced FTO-related decreases in stemness in HCT116 and HT29 CSCs. Berberine treatment also increased chemosensitivity in CSCs and promoted chemotherapy agent-induced apoptosis. Moreover, we also found that Berberine treatment increased FTO by decreasing β-catenin, which is a negative regulator of FTO.

**Conclusions:**

Our observation that Berberine effectively decreased m^6^A methylation by decreasing β-catenin and subsequently increased FTO suggests a role of Berberine in modulating stemness and malignant behaviors in colorectal CSCs.

## Introduction

Berberine hydrochloride (BBR), also known as Berberine, is a compound extracted from the traditional Chinese medicine Coptis chinensis (1). BBR has a wide range of pharmacological and therapeutic effects, and BBR has been widely used for its antimicrobial and antiprotozoal activities (2). Recently, as research continues, BBR has also been found to play a role in mood disorders (3), high blood pressure (4), hypercholesterolemia (5), hyperlipidemia (5), diabetes (6), heart failure (7), colorectal cancer (8), and other diseases. Because of its many effects, BBR is as commonly used as are aspirin and metformin. The study of BBR in colorectal cancer has made some progress, but few cases of its use have been reported in the literature. BBR inhibits the malignant behavior of colorectal cancer by targeting AMPK or the TGF-β1/Smad signaling pathway (9, 10), blocking the cell cycle, promoting the apoptosis of colorectal cancer cells, and inhibiting growth factor signaling pathways (11, 12).

A high-quality multicenter randomized, double-blind, controlled clinical study was conducted in seven hospitals in six provinces in China (13). A total of 1,136 patients were screened, and 1,108 patients with recently diagnosed colorectal adenomas who underwent total adenectomy were randomly assigned to two groups at a 1:1 ratio: the BBR group (553 patients, 0.3 g twice daily for 2 years) and the placebo group (555 patients). All patients were required to complete at least one colonoscopy during the follow-up period, which continued until recurrence of the adenoma was diagnosed or 2 years after the last patient was enrolled. Of the final 891 patients (429 in the BBR group and 462 in the placebo group), recurrence of colorectal adenomas was found during the follow-up colonoscopy in 155 patients (36%) in the BBR group and 216 patients (47%) in the placebo group. A total of 183 patients (43%) in the BBR group and 255 patients (55%) in the placebo group had polypoid lesions (including adenomas and serrated lesions) on follow-up colonoscopy. During the study period, 15 (3%) and 26 (6%) patients in the BBR and placebo groups developed advanced adenomas, respectively. The above data confirmed that BBR effectively reduced the risk of adenoma recurrence and the risk of recurrence of advanced adenomas and had a significant preventive effect on polypoid lesions.

Colorectal cancer stem cells (CSCs) are a dynamically changing subset of cells that are influenced by genomic, epigenetic, and microenvironmental factors, which were characterized by CD44 and CD133 (14, 15). CSCs have a self-renewal ability and unlimited proliferation and differentiation potential. Although these cells only account for a small portion of tumor cells, they are the key to the genesis and development of tumors. CSCs are highly resistant, proliferative, and metastatic, and even if only a small fraction survive, they can become the source of colorectal cancer recurrence. Therefore, we hope to explore the effect of BBR on CSC characteristics, including CSC proliferation, migration, invasion, and tumorigenesis, and to provide a theoretical basis for the clinical prevention of recurrence of colorectal cancer after radiotherapy and chemotherapy. According to a recent study, Relier and colleagues reported that m^6^A_m_ demethylation adjusts stem-like properties in colorectal cancer cells (16); this prompted us to investigate whether BBR affects stem-like properties *via* regulating the m6A methylation level.

In this study, we aimed to investigate the potential regulatory roles of Berberine in colorectal CSCs related to modification of m^6^A methylation.

## Material and Methods

### Cell Culture

HCT116 and HT29 cells were obtained from Feiouer company (Chengdu, China). The cells were cultured in Dulbecco’s modified Eagle’s medium (DMEM) with 10% fetal bovine serum and 1% penicillin–streptomycin. Cells were passaged every 3 days.

### Enrichment of Cancer Stem-Like Cells

In order to enrich CSCs *in vitro*, the cells were cultured in DMEM/F12 (D6434, Sigma) without serum (SF) and supplemented with 10 ng/ml basic FGF (F0291, Sigma), 2 ml glutamine, 20 ng/ml EGF (E9644, Sigma), 1% antibiotic–antifungal, and 1% B-27 supplement (17504044, Life Technologies).

To obtain singled CSCs from spheres, a SoniConvert^®^ Tissue Single-Cell Convertor (DocSense, Chengdu, China) was employed according to the manufacturer’s instruction. Briefly, spheres were cultured in digesting solution A for 10 min and homogenized for 3 s. After centrifugation, cells were suspended in medium.

### Cell Viability Assay

We used CCK-8 assay to detect the viability of cells. The cells were inoculated into a 96-well plate (5 × 10^3^ per well) and then placed overnight in a cell incubator at 37°C to make the cells stick to the wall. Ten, 20, and 40 μM of Berberine were used to treat the cells for 24 h. According to the proportion of 9:1, the culture medium and CCK-8 reagent were mixed and added to each well and placed in the incubator for 2 h, and the absorbance was determined at 450-nm wavelength using a enzyme-labeling instrument.

### Cell Cycle Distribution Analysis

Flow cytometry (FCM) was used to determine the effect of Berberine on the cell cycle. Cells were treated with 10, 20, and 40 μM of Berberine for 24 h and then fixed using 70% anhydrous ethanol overnight, stained with 50 μg/ml propidium iodide (PI, Sigma) for 30 min at 4°C, and then assessed with a BD FACSCanto II, BD Biosciences (San Jose, CA, USA). The cell phase is represented by G_0_-G_1_, S, and G_2_-M.

### Western Blot

1 × 10^6^ cells were suspended in 200 μl of RIPA buffer and lysed using the SoniConvert^®^ Tissue cell convertor (DocSense, Chengdu, China) following the manufacturer’s instruction. The protein concentration was measured by BCA protein assay (Sigma). The protein was loaded into a 10% SDS-PAGE and transferred to a PVDF membrane. The membrane was then incubated with the respective primary including Cyclin D1 (cat. no. ab16663), p27 (cat. no. ab32034), p21 (cat. no. ab109520), β-actin (cat. no. ab8226), CD44 (cat. no. ab189524), CD133 (cat. no. ab222782), METTL3 (cat. no. ab195352), METLL14 (cat. no. ab220030), YTHDF1 (cat. no. ab252346), WTAP (cat. no. ab195380), FTO (cat. no. ab126605), ALKBH5 (cat. no.), PARP (cat. no. ab191217), cleaved-PARP (cat. no. ab32064), cleaved-caspase 3 (cat. no. ab32042) at dilution of 1:1,000, and secondary antibodies, including anti-rabbit secondary antibody (cat. no. ab6747) at dilution of 1:5,000. Finally, protein signals were detected by a chemiluminescence kit (Thermo Scientific, USA).

### Annexin V/PI Double Staining for Detecting Apoptosis

At 48 h after dosing, the intervention cells and control cells were treated with trypsin and washed with PBS (0.15 mol/l, pH 7.2) for two times. The cells were centrifuged at 3,000 r/min for 5 min, then the supernatant was discarded and the pellet was resuspended in 1× binding buffer at a density of 1.0 × 10^5^–1.0 × 10^6^ cells per mL. One hundred microliters of the sample solution was transferred to a 5-ml culture tube and incubated with 5 µl of FITC-conjugated Annexin V and 5 µl of PI (BD Biosciences, Franklin Lakes, NJ, USA) for 15 min at room temperature in the dark. Four hundred microliters of 1 × binding buffer was added to each sample tube, and the samples were analyzed by FACS using CellQuest Research Software.

### Animal Experiments

All the animal experiments were conducted according to the ethics committee of the Institutional Animal Care and Use Committee of Institute of Chengdu University of Traditional Chinese Medicine. Four-week-old female BALB/c nude mice were purchased from Dashuo Experimental Animal Company (Chengdu, China) and raised in the SPF animal facilities.

5 × 10^5^ HCT116 CSCs were subcutaneously injected into the mice similarly as nude mice. Seven days later, 5, 10, or 20 mg/kg Berberine was intraperitoneally injected. The same volume of PBS was injected and considered as negative control. For each group, n = 5. Mouse weight and tumor size were measured every 7 days after injection.

### Detection of m^6^A Level

Total mRNA was extracted from tissue samples using TRIzol reagent (Thermo Scientific, USA), as described previously (16). An m^6^A RNA methylation quantification kit (Thermo Scientific, USA) was purchased for directly detecting the m6A RNA level using total mRNA. The percentage of m6A-modified mRNA in the total mRNA (m6A%) was used to evaluate the mRNA m6A level in this study. In brief, according to the manufacturer’ s protocol, 200 ng mRNA from each sample was allocated by pipette into assay wells. Subsequently, a capture antibody specific for m6A (Synaptic Systems, catalog no. 202003, at dilution of 1:2,000) was added to the wells. After washing, a detection antibody (Abcam, catalog no. ab6747, at dilution of 1:5,000) was added to the wells. The developer solution was added to each well following the wash steps to remove any liquid while protecting samples from light. The color development was arrested, and the intensity of color was measured at 450-nm wavelength. The proportion of m6A in total mRNA was calculated as a percentage according to the standard curve.

### Clinical Colorectal Cancer Tissue Microarray

Liver tissue microarrays (HColA160CS01) were purchased from Outdo Biotech (Shanghai Outdo Biotech Co., Ltd., China), which contained paired COAD and adjacent tissues from 80 COAD patients. Completed clinicopathology data were collected for further analysis. The EnVision+detetion system (Dako) was employed to perform immunohistochemistry following the manufacturer’s instructions. A semiquantitative scoring criterion for IHC of FTO staining was used (week or moderated was considered as negative; strong was considered as positive). Two independent pathologists, blinded to the clinic pathological information, performed the identification.

### Transfection of Lentivirus or shRNA

To knock down an inverted and self-complementary hairpin DNA oligonucleotide encoding, a short-hairpin RNA targeting β-catenin mRNA was chemically synthesized (RiboBio, Guangzhou, China), aligned, and cloned into the lentiviral vector pLL3.7 (RiboBio, Guangzhou, China) that co-express the fluorescent protein GFP. As a control, we used shRNA targeting Luciferase mRNA. Oligos used to construct the shRNA targeting mouse a were 5′-TGGTGCTGCTATGTCAAATGCAAGATTCAAGAGATCTTGCATTTGACATAGCAGCACCTTTTTTC-30; 5′-TCGAGAAAAAAGGTGCTGCTATGTCAAATGCAAGATCTCTTGAATCTTGCATTTGACATAGCAGCAC-3′ (reverse). Oligos used as control shRNA were 5′-TGTTCTCCGAACGTGTCACGTTTCAAGAGAACGTGACACGTTCGGAGAACTTTTTTC-3′ (forward); 5′-TCGAGAAAAAAGTTCTCCGAACGTGTCACGTTCTCTTGAAACGTGACACGTTCGGAGAACA-3′ (reverse).

### Real-Time Quantitative PCR

Total RNA was extracted using the TRIzol reagent (Life Technologies, Grand Island, NY, USA) according to the manual. After RNA isolation, the concentration of purified RNA was determined by the UV spectrophotometer (Life Technologies, Grand Island, NY, USA). cDNA was reversibly transcribed from the extracted total RNA using a Reverse Transcriptase Kit (RiboBio, Guangzhou, China). For analyzing mRNA, SYBR Green Master Mix (Life Technologies, Grand Island, NY, USA) was employed in a ABI 7500 system (Applied Biosystems, Foster City, CA, USA) under the following conditions: 95°C 10 min, 60 cycles of 95°C 15 s, and 60°C 1 min. The specific primers used were as follows: β-actin forward: 5′-CATGTACGTTGCTATCCAGGC-3′; reverse: 5′-CTCCTTAATGTCACGCACGAT-3′; p21 forward: 5′-TGTCCGTCAGAACCCATGC-3′; reverse: 5′-AAAGTCGAAGTTCCATCGCTC-3′; cyclin D1 forward: 5′-GCTGCGAAGTGGAAACCATC-3′; reverse: 5′-CCTCCTTCTGCACACATTTGAA-3′; p27 forward: 5′-AGGAGGAGATAGAAGCGCAGA-3′; reverse: 5′-GTGCGGACTTGGTACAGGT-3′; METTL3 forward: 5′-TTGTCTCCAACCTTCCGTAGT-3′; reverse: 5′-CCAGATCAGAGAGGTGGTGTAG-3′; METTL14 forward: 5′-AGTGCCGACAGCATTGGTG-3′; reverse: 5′-GGAGCAGAGGTATCATAGGAAGC-3′. YTHDF1 forward: 5′-ACCTGTCCAGCTATTACCCG-3′; reverse: 5′-TGGTGAGGTATGGAATCGGAG-3′. WTAP forward: 5′-CTTCCCAAGAAGGTTCGATTGA-3′; reverse: 5′-TCAGACTCTCTTAGGCCAGTTAC-3′. FTO forward: 5′-ACTTGGCTCCCTTATCTGACC-3′; reverse: 5′-TGTGCAGTGTGAGAAAGGCTT-3′. ALKBH5 forward: 5′-CGGCGAAGGCTACACTTACG-3′; reverse: 5′-CCACCAGCTTTTGGATCACCA-3′.

### Invasion Assay

Cell invasion was examined using a 24-well Transwell insert system (Corning, NY). For invasion assay, 1 × 10^4^ cells were plated in the top chamber containing the Matrigel-coated membrane. Each well was freshly coated with Matrigel (60 μg; BD Biosciences). Cells were plated in medium without serum or growth factors, and the medium supplemented with DMEM and 10% FBS was used as a chemoattractant in the lower chamber. The cells were incubated for 48 h. Cells on the lower surface of the membrane were fixed with methanol and stained with crystal violet. The number of cells invading through the membrane was counted under a microscope (Olympus, Tokyo, Japan). The invasion rate was calculated from five fields under random selection.

### Statistical Analysis

Each experiment was performed at least three times. The software GraphPad Prism software was used for data analysis. Statistical analyses were performed using ANOVA (equal variance) or Welch’s ANOVA (unequal variance). A statistically significant difference among groups was defined as p < 0.05.

## Results

### Berberine Inhibit Malignancies of CSCs Derived From HCT116 and HT29

CSCs play a pivotal role in various key oncogenic processes including tumor initiation, recurrence, metastasis, and chemoresistance (17, 18). To investigate the effect of Berberine on CRC-derived stem-like cells, we enriched spheres from HCT116 and HT29 cells by maintaining them in ultra-low-attachment dishes in serum-free and stem cell-inducing medium (DMEM/F12 supplemented with B27, EGF, and bFGF) (**Figure 1A**). We also noted an upregulation of stemness-related cell markers CD44 and CD133, in spheres compared to those in parental cells (**Figure 1B**), which confirmed the successful enrichment of CSCs from HCT116 and HT29 cells. The obtained spheres were then used as a model system to further investigate the effects of Berberine on CSCs.

**Figure 1:** Berberine inhibited malignancies and induced apoptosis in HCT116 and HT29 CSCs. **(A)** Parental HCT116 and HT29 cells were cultured in serum-free medium for 14 days, and spheres were obtained. **(B)** CD44 and CD133 protein levels were detected by performing the Western blot in total protein. **(C)** By being cocultured with 10, 20, or 40 μM of Berberine for 1 to 5 days, cell viability was measured by performing CCK-8 assay. p < 0.05, *vs.* mock group. By being cocultured with 10, 20, or 40 μM of Berberine for 24 h, cell cycle distribution was analyzed by performing flow cytometry assay **(D)** and p21, p27, and Cyclin D1 protein levels were measured by performing Western blot **(E)**. p < 0.05, *vs.* mock group. **(F)** Tumor formation ability of CSCs was measured by being cocultured with 10, 20, or 40 μM of Berberine for 14 days. **(G)** By being cocultured with 10, 20, or 40 μM of Berberine for 24 h, cell apoptosis was measured by performing Annexin V-FITC/PI double staining. *P < 0.05, vs. mock group.

When we cultured singled cells obtained from spheres in the presence of 10, 20, or 40 μM of Berberine for 5 days, we observed a significant decrease in the cell viability on a dose-dependent manner in both two cell cultures (**Figure 1C**). After a 24-h treatment of 10, 20, or 40 μM of Berberine, cell-cycle distribution was then analyzed, and results presented that Berberine treatment significantly increased the proportion of G_1_/G_0_ and decreased that of G_2_^/^M (**Figure 1D**). To clarify the mechanism of Berberine involved in cell-cycle arrest, we characterized the expression of G1-phase checkpoint proteins p21 and p27 and expectedly observed that Berberine significantly increased the p21 and p27 protein levels (**Figure 1E**). Decreased cyclin D1 by Berberine treatment was also observed, which indicated that Berberine may induce cell-cycle arrest by inhibiting G_1_-to-S transition (**Figure 1E**). We also accessed tumor formation ability with the presence of Berberine, and expectedly, we observed that Berberine obviously decreased tumor formation ability in soft agar (**Figure 1F**). By performing apoptosis assay, it was also observed that 40 μM of Berberine treatment significantly induced apoptosis (**Figure 1G**).

### Berberine Increased FTO and Decreased m6A Modification in Total RNAs

Dynamic m^6^A modification of total RNAs plays key roles in regulating malignancies in several cancers, including self-renewal capacity and maintenance of stemness (19–21), and leads us to further investigate the potential role of Berberine treatment on m6A modification in colorectal CSCs. We firstly compared the mRNA expression of m^6^A modification-related genes, including METLL3, METLL14, YTHDF1, WTAP, FTO, and ALKBH5 between cancer and normal samples. The results indicated that METTL3 and ALKBH5 were significantly downregulated, while WTAP and YTHDF1 were significantly upregulated in cancer samples (**Figure 2A**). We then measured protein levels of METLL3, METLL14, YTHDF1, WTAP, FTO, and ALKBH5 (**Figure 2B**). To determine the changes in the level of m^6^A during Berberine treatment, we measured the level of m^6^A in CSCs that were exposed to Berberine for 14 days. We found that the level of m^6^A was significantly decreased in Berberine-treated cells (**Figure 2C**), and mRNA, protein level of m^6^A demethylases, and FTO were significantly upregulated (**Figures 2D, E**). This indicated that Berberine potentially decreased the m^6^A modification of total RNAs *via* upregulating FTO.

**Figure 2:** Berberine decreased m6A modification of total RNAs in CSCs. **(A)** METLL3, METLL14, FTO, WTAP, YTHDF1, and ALKBH5 mRNAs were analyzed in colorectal cancer samples compared with normal samples. **(B)** Protein levels of METLL3, METLL14, FTO, WTAP, YTHDF1, and ALKBH5 in CSCs and parental cells were measured by performing western blot. *p < 0.05, *vs.* PCs. **(C)** Total m^6^A levels in CSCs with or without Berberine treatment by EpiQuik m6A RNA Methylation Quantification Kit. RT-qPCR testing the mRNA levels **(D)** and Western blot examine the protein levels **(E)** of m^6^A regulating proteins. *p < 0.05, **p < 0.01, *vs.* 0 μM treat.

To clarify the relationship between malignancies and FTO protein levels in COAD, we used COAD tissue microarray to investigate the correlation in the clinic. Tissue sections of 80 COAD patients were subjected to IHC analysis. Full-scale scanning of tissue microarray was shown as indicated (**Figure 3A**), with representative images under high-power field microscopy (**Figure 3B**). Intriguingly, semiquantified analyses clearly revealed that in II–III phases and III phase cancer cases, the positive rate is approximately 70% (7/10) and 66.7% (6/9), which are higher than that in total cases (28/80) (**Figure 3C**). This result indicated that FTO may be positively related to malignancies and poor prognosis in COAD patients.

**Figure 3:** FTO expression was identified in clinical COAD patients. **(A)** Clinical COAD tissue microarray assay was analyzed by IHC with anti-FTO antibody, and full scan of tissue microarray is shown as indicated. **(B)** Representative images of FTO staining under high power field (HPF) from clinical COAD tissue microarray. **(C)** Qualitative analysis for expression pattern and stained grade of FTO in clinical COAD tissue microarray.

### Berberine Regulated Stemness and Malignancies of HCT116 CSCs

To investigate the effect of Berberine on CSC stemness, HCT116 CSCs were cocultured with 40 μM of Berberine for 14 days, and formed spheres were imaged (**Figure 4A**). It was observed that addition of Berberine inhibited sphere formation, which was reversed by inhibition of FTO by adding FB23-2. Consistently, CD44 and CD133 were decreased by Berberine treatment which was reversed by addition of FB23-2 (**Figure 4B**). To confirm the role of FTO on m^6^A modification, we knocked down FTO in HCT116 CSCs by infecting the lentivirus-coding shRNA target to FTO mRNA efficiently (**Figures 4C, D**) and then detected the level of m^6^A methylation. The results showed that the decrease in m^6^A methylation was reversed by FTO knockdown and FTO inhibition by addition of FB23-2, a potent and selective inhibitor of FTO (**Figure 4E**). We also introduced FTO-expressing lentivirus and efficiently overexpressed FTO in HCT116 CSCs (**Figures 4F, G**) and found that Berberine treatment and overexpressed FTO presented similar effects on m6A methylation (**Figure 4H**).

**Figure 4:** Berberine regulated m6A methylation and sphere formation *via* regulating FTO. **(A)** With the addition of 40 μM of Berberine, sphere formation of HCT116 was observed after a 14-day culture. **(B)** Western blot was performed to detect CD44 and CD133 protein levels in HCT116 CSCs. *p < 0.05, *vs.* mock group; ^#^p < 0.05, *vs.* BER/vehicle group. Lentivirus containing shRNA coding sequence target to FTO mRNA was efficiently transfected into HCT116 CSCs **(C)** and efficiently knockdown FTO protein **(D)**. **(E)** Total m^6^A levels in HCT116 CSCs were measured. *p < 0.05, *vs.* mock group; ^#^p < 0.05, *vs.* shScrambled group; ^&^p < 0.05, *vs.* mock group. FTO was efficiently transfected into HCT116 cells **(F, G)**. **(H)** Total m^6^A levels in HCT116 CSCs were measured. *p < 0.05, *vs.* mock group; ^#^p < 0.05, 20 μM Berberine-treated group.

We then confirmed whether the effect of Berberine on malignancies is *via* upregulated FTO or not. As is shown in **Figure 5A**, expectedly, G1 phase block was induced by Berberine treatment and FTO overexpression, which were reversed by adding FB23-2 (**Figures 5A, B**). We also measured invasive ability after FTO addition. Expectedly, inhibition of FTO induced by Berberine promoted invasive ability which was inhibited by Berberine (**Figure 5C**).

**Figure 5:** Berberine blocked the cell cycle *via* upregulating FTO. The effects of Berberine on cell cycle distribution *via* FTO were confirmed by performing PI staining followed by flow cytometry **(A, B)**. *p < 0.05, *vs.* mock group; ^#^p < 0.05, *vs.* BER/vehicle group. **(C)** Transwell assay was performed to detect invasive assay.

To further confirm the inhibitory effect of Berberine on HCT116 CSC growth *in vivo*, xenograft-transplanted mice were intraperitoneally injected using 5, 10, or 20 mg/kg 5 days a week. Expectedly, administration of Berberine inhibited tumor growth *in vivo* than the mock group, without disturbing the body weight (**Figures 6A, B**). Proliferation marker (Ki-67) was not significantly decreased in nude mice (**Figures 6C, D**). Taken together, our *in vivo* data indicate that administration of Berberine in CSCs inhibited tumor growth *in vivo*.

**Figure 6:** Berberine inhibited *in vivo* tumor formation ability. **(A)** Volume of CSCs formed tumors in nude mice after seeding 5 × 10^5^ cells. **(B)** Weight of nude mice and size of seeded tumors were measured at 7, 14, 21, and 28 days after transplantation. *p < 0.05, *vs.* mock group. Tumor formation was morphologically identified by H&E staining **(C)**, and cell proliferation marker Ki-67 **(D)** were further measured.

### Berberine Enhanced Chemosensitivity *via* Regulating FTO

Previous reports presented that Berberine enhances chemosensitivity and induces apoptosis in various cancer cells (22, 23) and prompted us to extend these findings to chemoresistance, another hallmark of CSC. FIRI (50 μM 5-fluorouracil (5-FU) +500 nM SN38, an active metabolite of irinotecan), which was employed to treat metastatic colorectal cancer (24), was employed. Berberine pretreatment for 72 h conferred significant chemo-promoting effects on HCT116 and HT29 CSCs, which were reversed by addition of FB23-2 (**Figure 7A**). Next, we performed Annexin V-FITC/PI double staining followed by flow cytometry to detect the apoptotic rate and observed that Berberine pretreatment significantly increased the FIRI chemosensitivities of both HCT116 and HT29 cells (**Figure 7B**). We also confirmed the promoted apoptotic rate in these cells by the use of the Western blot (**Figure 7C**). Above all, these results support a role for Berberine in sensitizing HCT116 and HT29 CSCs to FIRI treatment.

**Figure 7:** Berberine promoted chemosensitivity. **(A)** Sulforhodamine B assay was performed to measured the toxicity of FIRI to HCT116 and HT29 CSCs. *p < 0.05, *vs.* mock group; ^#^p < 0.05, *vs.* Berberine-treated group. **(B)** Annexin V-FITC/PI double staining was performed followed by flow cytometry to measure the apoptotic rate. *p < 0.05, *vs.* mock group; ^#^p < 0.05, *vs.* Berberine-treated group. **(C)** Western blot was performed to detect apoptosis hallmarkers, cleaved PARP, and cleaved caspase-3.

### Berberine Regulated Mitochondrial ATP Synthesis Partially *via* Regulating FTO

It is reported that Berberine targets mitochondrial dysfunction and aberrant cellular energetic metabolism (25). We hypothesized that Berberine, at least partially, regulates energetic metabolism *via* FTO, which restores mitochondrial activity *via* transcriptionally activating PGC-1α (26). To confirm whether Berberine regulates mitochondrial energetic metabolism *via* upregulating FTO, HCT116 CSCs were treated with Berberine with or without an FTO inhibitor, FB23-2, for 1, 3, or 7 days. Expectedly, PGC-1α was transcriptionally and posttranscriptionally upregulated after 1 and 3 days (**Figures 8A, B**). Addition of FB23-2 reversed the upregulation of PGC-1α, indicating that Berberine upregulated PGC-1α, *via* activating the FTO axis. Although the effect of Berberine on mitochondrial DNA content presented a reversible tendency, its effect on energetic metabolism presented after long-term treatment (**Figures 8C, D**).

**Figure 8:** Berberine regulated mitochondrial energy metabolism partially *via* upregulating FTO. After being treated by BER or BER/FB23-2 for 1, 3, or 7 days, PGC-1α mRNA **(A)**, protein level **(B)**, mitochondrial DNA content **(C)**, and mitochondrial ATP synthesis **(D)** were measured. *p < 0.05, *vs.* mock group; *p < 0.05, *vs.* BER group.

### Berberine Regulated FTO *via* Downregulating β-Catenin

Berberine was reported to antagonize the Wnt/β-catenin axis in colon cancer *via* inducing β-catenin proteasomal degradation involving retinoid X receptor α (27), which prompted us to confirm whether Berberine affects β-catenin expression in HCT116 and HT29 CSCs. After 12 and 24 h treatment using 10, 20, and 40 μM of Berberine, Berberine treatment significantly decreased β-catenin expression (**Figure 9A**), without disturbing β-catenin mRNA levels (**Figure 9B**). A decrease of β-catenin by Berberine treatment for 24 h significantly decreased the mRNA and protein levels of Cyclin D1 and Axin2 (**Figure 9C**), which are two β-catenin target genes (28, 29). This further confirmed the effects of Berberine on β-catenin transcriptional activity.

**Figure 9:** Berberine decreased β-catenin and its downstream target genes. **(A)** After 12 or 24 h treatment using 10, 20, and 40 μM of Berberine, β-catenin protein levels were measured by Western blot in both HCT116 and HT29 CSCs. *p < 0.05, *vs.* mock group at 12 h; ^#^p < 0.05, *vs.* mock group at 24 h. **(B)** After 12 or 24 h treatment using 10, 20, and 40 μM of Berberine, β-catenin mRNA levels were measured by RT-qPCR. After 40 μM of Berberine treatment, Axin2 and Cyclin D1 protein levels were measured by Western blot and RT-qPCR (C&D). *p < 0.05, *vs.* mock group; ^#^p < 0.05, *vs.* mock group. After 40 μM of Berberine treatment, Axin2 and Cyclin D1 protein levels were measured by Western blot and RT-qPCR **(C, D)**. *p < 0.05, vs. mock group; ^#^p < 0.05, vs. mock group.**P < 0.01, vs. mock group at 24 h.

β-Catenin transcriptionally inhibited FTO by binding to its promoter region (30), which made us hypothesize that Berberine treatment upregulated FTO *via* downregulating β-catenin. Treatment of Berberine expectedly upregulated FTO mRNA and was reversed by addition of 60 ng/ml Wnt 3a (**Figure 10A**). Knockdown of β-catenin expectedly upregulated FTO mRNA, which was confirmed by detecting β-catenin and FTO protein levels (**Figure 10B**).

**Figure 10:** Berberine upregulated FTO *via* downregulating β-catenin. After Berberine treatment, activating wnt signaling or knockdown β-catenin for 48 h, FTO mRNA levels **(A)** and protein levels **(B)** were measured. *p < 0.05, *vs.* mock group; ^#^p < 0.05, *vs.* Berberine-treated group; ^&^p < 0.05, *vs.* shScrambled group.

## Discussion

Colorectal cancer therapies frequently fail due to the existence of cancer stem-like cells (CSCs). Thus, novel CSC-targeting or CSC-sensitizing antitumor drugs appear to be a plausible means to enhance the antitumor effects in CRC. Being used increasingly in the clinic, traditional Chinese medicine (TCM) has been found to be a promising alternative therapeutic option for CRC, in addition to surgery and chemotherapy (31). Solid evidence demonstrated that TCM administration efficiently inhibited malignant behaviors in CRC (32) and promoted the survival of CRC patients (33), which is increasingly important and necessary for the investigation of the underlying mechanisms of the antitumor roles of TCM, especially their components. Berberine, a natural plant alkaloid extracted from the TCM herb Coptis chinensis, has been shown to play antitumor roles in several kinds of cancers, including CRC (34) and liver, breast (35), prostate (36), and lung (37) cancers. In particular, in CRC therapy clinics, Berberine administration was proven to be safe and effective in reducing the risk of recurrence of colorectal adenoma, and it was an option for chemoprevention after polypectomy (13). Considering that the existence of colorectal CSCs remarkably contributes to recurrence and metastasis (38), in our current study, we generated *in vitro* and *in vivo* data to investigate the antitumor effects of Berberine in colorectal CSCs. Furthermore, we investigated the potential mechanisms.

Previous studies have shown that fat mass and obesity-associated protein (FTO) impact the stemness of CSCs in colorectal cancer by exerting its N^6^,2′-O-dimethyladenosine (m^6^A_m_) demethylase activity (16). After Berberine treatment, FTO was transcriptionally upregulated in HCT116 and HT29 CSCs in a dose-dependent manner (**Figures 3B, D**). As expected, m^6^A modification was decreased after Berberine treatment (**Figure 3C**). METTL3 and METTL14 (methyltransferase-like proteins) form the core heterodimeric complex of m6Ase along with the scaffold protein WTAP (Wilm’s tumor-associated protein), whereas FTO and ALKBH5 reverse methylation (39). Interestingly, Berberine treatment slightly affected METLL3, METLL14, YTHDF1, WTAP, and ALKBH5 levels, indicating that Berberine affects m^6^A modification specifically by regulating FTO. Global m^6^A modification was found to be critical for maintaining stemness in cancer stem-like cells (39), which prompted us to question whether Berberine-induced FTO upregulation affects the characteristics of colorectal CSCs. As expected, both upregulation of FTO by Berberine treatment and exogenous overexpression decreased sphere formation and stem cell markers in HCT116 and HT29 CSCs. The addition of FB23-2, a small molecule that binds specifically to FTO and thus induces FTO depletion, reversed the effect of Berberine on sphere formation, further supporting that Berberine modified stemness *via* effects on FTO-related m6A methylation but not on METLL3, METLL14, YTHDF1, WTAP, or ALKBH5. According to the recent usage of single-cell multi-omics and spatial transcriptomics (40–42), which present more insight into the effects of BER on m6A methylation, it is worth performing this analysis in further investigation.

In colorectal cancer, aberrant activation of the Wnt/β-catenin signaling pathway is one of the main causes of colon tumorigenesis and metastasis (43). Ruan and colleagues reported that in colon cancer cells, Berberine binds retinoid X receptor alpha (RXRα) and subsequently suppresses β-catenin signaling by inhibiting β-catenin transcription (27). It has also been reported that Berberine represses β-catenin translation involving 4E-BPs in hepatocellular carcinoma cells by activating AMP-activated protein kinase (AMPK) (9). As expected, in HCT116 and HT29 CSCs, Berberine treatment significantly decreased β-catenin protein levels without disturbing the mRNA levels (**Figures 8A, B**). This result demonstrated that Berberine treatment affects β-catenin posttranscriptionally, which is consistent with previous findings (9, 27). Inactivation of the Wnt/β-catenin signaling pathway decreased the expression of downstream target genes, including Axin2 and cyclin D1. Downregulation of β-catenin increased FTO protein levels, which presented a similar effect to that seen in the β-catenin knockdown group. Taken together, these data indicated that Berberine decreased β-catenin and thus increased the FTO protein levels.

## Conclusion

Our study demonstrates that Berberine regulates the stemness of CSCs by inhibiting β-catenin and its downstream signaling partners, especially FTO, in HCT116 and HT29 CSCs. This pathway also seems to mediate Berberine-associated tumor regulation. Some limitations of this study include the *in vitro* cell experiments. Our results identify Berberine as a novel m6A methylation modulator that induces promising therapeutic effects in colon cancer by targeting CSCs, and our findings provide new strategies for the design of new Wnt/β-catenin-based antitumor agents and drug combinations.

## Data Availability Statement

The original contributions presented in the study are included in the article/**Supplementary Material**. Further inquiries can be directed to the corresponding authors.

## Ethics Statement

The animal study was reviewed and approved by the Institutional Animal Care and Use Committee of Institute of Chengdu University of Traditional Chinese Medicine.

## Author Contributions

ZZ, JZ, QG, JT, and QH designed the experiments and performed most of the experiments included in this study. KP and YY performed the experiments on processing cells. ZZ, NC, GZ, and MZ are responsible for data collection and performed the statistical analysis. ZZ and QZ performed the molecular experiments. ZZ and QH wrote the manuscript. JT revised the manuscript. All authors contributed to the article and approved the submitted version.

## Funding

This work was supported by The General Program (Key Program, Major Research Plan) of the National Natural Science Foundation of China http://isisn.nsfc.gov.cn/egrantweb/ (No. 82074298).

## Conflict of Interest

The authors declare that the research was conducted in the absence of any commercial or financial relationships that could be construed as a potential conflict of interest.

## Publisher’s Note

All claims expressed in this article are solely those of the authors and do not necessarily represent those of their affiliated organizations, or those of the publisher, the editors and the reviewers. Any product that may be evaluated in this article, or claim that may be made by its manufacturer, is not guaranteed or endorsed by the publisher.
